# miR-195-5p/NOTCH2-mediated EMT modulates IL-4 secretion in colorectal cancer to affect M2-like TAM polarization

This article has been retracted.

**DOI:** 10.1186/s13045-019-0708-7

**Published:** 2019-02-26

**Authors:** Xiaobin Lin, Shuyi Wang, Min Sun, Chunxiao Zhang, Chen Wei, Chaogang Yang, Rongzhang Dou, Qing Liu, Bin Xiong

**Affiliations:** 1 Department of Gastrointestinal Surgery, Zhongnan Hospital of Wuhan University, No.169 Donghu Road, Wuchang District, Wuhan, 430071 China; 2 Department of Gastric and Colorectal Surgical Oncology, Zhongnan Hospital of Wuhan University, No.169 Donghu Road, Wuchang District, Wuhan, 430071 China; 3 Hubei Key Laboratory of Tumor Biological Behaviors, No.169 Donghu Road, Wuchang District, Wuhan, 430071 China; 4 Hubei Cancer Clinical Study Center, No.169 Donghu Road, Wuchang District, Wuhan, 430071 China; 5 Department of General Surgery, Taihe Hospital, Hubei University of Medicine, Shiyan, 442000 China

**Keywords:** miR-195-5p, NOTCH2, CRC, EMT, IL-4, TAMs

## Abstract

**Background:**

Tumor microenvironment (TME) is a complex environment containing tumor cells, tumor-associated macrophages (TAMs), interstitial cells, and non-cellular components. Epithelial–mesenchymal transition (EMT), as a major actor in cancer tumorigenicity and metastasis, was involved in the interaction between TAMs and tumor cells. However, the potential mechanisms of EMT and how EMT-programmed tumor cells affect M2-like TAMs still need further exploration.

**Methods:**

An integrated analysis of nine CRC miRNA expression datasets was performed. Functional assays, including the EdU, clone formation, wound healing, and transwell assays, were used to determine the anticancer role of miR-195-5p in human CRC progression. Furthermore, RNA immunoprecipitation, RNA decay, and dual-luciferase reporter assays were used to determine the mechanism of miR-195-p CRC progression. Then co-culture, migration, and ELISA assays were applied to determine the role of miR-195-5p in macrophage recruitment and alternative polarization. Xenograft mouse models were used to determine the role of miR-195-5p in CRC tumorigenicity and TAM polarization in vivo.

**Results:**

An integrated analysis confirmed that miR-195-5p was significantly downregulated in CRC tissues, and patients with a low level of miR-195-5p had significantly shortened overall survival as revealed by the TCGA-COAD dataset. Altered miR-195-5p in colon cancer cells led to distinct changes of proliferation, migration, invasion, and EMT. Mechanistically, miR-195-5p regulated NOTCH2 expression in a post-transcriptional manner by directly binding to 3′-UTR of the Notch2 mRNA. Subsequently, miR-195-5p/NOTCH2 suppressed GATA3-mediated IL-4 secretion in CRC cells and ultimately inhibited M2-like TAM polarization.

**Conclusions:**

miR-195-5p may play a vital role in regulating NOTCH2-mediated tumor cell EMT, thereby affecting IL-4-related M2-like TAM polarization in CRC.

**Electronic supplementary material:**

The online version of this article (10.1186/s13045-019-0708-7) contains supplementary material, which is available to authorized users.

## Background

Metastasis is an important step in the development of tumors and causes poor prognosis [1]. Epithelial–mesenchymal transition (EMT), as a major actor modulating tumor metastasis [2, 3], may be involved in the interaction between the tumor cells and tumor microenvironment (TME) [2, 4]. EMT-programmed tumor cells could secrete amounts of inflammatory mediators to change cellular and non-cellular components in TME [5–8]. As the most abundant immune cells in TME, tumor-associated macrophages (TAMs) can respond to various factors produced by tumor cells in the TME [9, 10]. EMT-programmed tumor cells can secrete mediators to activate TAMs to M2 phenotype [10], thereby facilitating tumor progression and metastasis [11–14]. Although the interplay between tumor cells and macrophages has been established, the understanding of EMT tumor cells modulating TAM polarization is limited.

Multiple signaling pathways cooperate in the initiation and progression of EMT [15]. Recent studies have showed that the Notch pathway was involved in tumor EMT [16–20]. NOTCH2, as one of the NOTCH receptors, is a single-pass transmembrane receptor activated by ligands of the DSL (Delta-like and Jagged) family in humans. Ligand binding to the extracellular domain of NOTCH2 induces release of the NOTCH2 intracellular domain (N2ICD; activated NOTCH2). Then N2ICD translocates to the nucleus, where it binds the transcription factor RBPJ, resulting in the complex activation of target genes related to EMT [18]. In addition, the Notch pathway activation was necessary in GATA3-induced IL-4 secretion [21, 22], which was widely accepted to activate M2-like macrophages [23]. It indicated that the Notch pathway plays pivotal roles in tumor EMT and macrophage alternative polarization in TME. However, whether the NOTCH pathway promotes CRC EMT to affect TAM polarization is still incompletely understood.

MicroRNAs (miRNAs) are a large class of small non-coding RNAs, which regulated the expression of mRNAs by binding the 3′-untranslated regions (3′-UTRs) or amino acid coding sequences [9]. miR-195-5p as a member of the miR-15/107 family has been widely explored in various cancers and was considered as a tumor suppressor to inhibit proliferation [24] and enhance radiochemosensitivity [25, 26] in CRC [12]. We had demonstrated that miR-195-5p is a suppressor of YAP1 in colorectal cancer EMT. However, how miR-195-5p-mediated EMT modulates cytokine secretion in CRC to affect TAM polarization is unclear. Taking into account that NOTCH2 may be a target of mR-195-5p, we hypothesized that miR-195-5p/NOTCH2 may influence CRC EMT status and modulate IL-4 mediated M2-like TAM polarization.

In this study, we performed an integrated analysis with nine datasets and identified miR-195-5p deregulation in primary tumors compared to paired adjacent normal tissue (ANT). A high level of miR-195-5p in patients was with favorable survival. In vitro and in vivo experiments have showed that aberrant expression of miR-195-5p could significantly reduce proliferation, migration, invasion, and EMT, confirming its anti-tumor functions. We further revealed that miR-195-5p inhibited NOTCH2 expression in a post-transcriptional manner, leading to downregulation of GATA3 and IL-4, ultimately suppressing M2-like TAM polarization. These observations highlighted the role of miR-195-5p/NOTCH2-mediated CRC EMT in TAM alternative polarization.

## Materials and methods

Detailed materials and methods are provided in supplemental experimental procedures (Additional file 1).

### Patient samples

For this study, we collected 30 paired CRC samples and ANT (distance to cancer > 5 cm) from patients who had been diagnosed with primary CRC by pathological assessment of tissues and undergone surgeries with complete prognostic information at the Zhongnan Hospital of Wuhan University between January 2016 and July 2018. No any neoadjuvant radiotherapy or/and chemotherapy was managed. The study was endorsed by the Research Ethics Committee of Wuhan University (Wuhan, Hubei, PR China). Informed consents were obtained from all participating patients.

### Cell lines

The normal intestinal epithelium cell line NCM460 and CRC cell lines (DLD-1, HCT116, SW480, SW620, HCT116, and HT29) were obtained from the Cell Bank of Wuhan University. The monocyte cell line was purchased from ATCC. Cells were cultured in RPMI 1640 medium (Invitrogen, Shanghai, China) containing 10% heat-inactivated (56 °C, 30 min) fetal calf serum, streptomycin (100 U/mL), and penicillin (100 U/mL), and maintained in a humidified atmosphere of 5% CO_2_ at 37 °C.

### Transfection of miR-195 mimic, inhibitor, and siRNA of the target gene

Hsa-miR-195 mimic and mimic negative control (NC), hsa-miR-195 inhibitor, and inhibitor negative control (NC) were purchased from RiboBio (Guangzhou, China). NOTCH2 siRNAs (Notch2-homo-1815, 2501 and 3130) were purchased from GenePharma (Shanghai, China). Cells were cultured in complete medium at least 24 h before transfection. Cells were washed with phosphate-buffered saline (PBS, pH 7.4) before transient transfection. Transfections were performed by Lipofectamine 2000 (Invitrogen, USA) according to the manufacturer’s protocol with RNA oligonucleotides at a final concentration of 50 nM.

### RNA immunoprecipitation (RIP) assay

RIP was performed using the Magna RIP RNA-Binding Protein Immunoprecipitation Kit (Millipore, MA, USA) according to the manufacturer’s protocol. In short, 5 × 10^7^ cells were lysed in polysome lysis buffer for each group. The expression of AGO2 protein was detected by western blotting, and then the supernatant was immunoprecipitated with antibody to AGO2 with protein A/G magnetic beads at 4 °C overnight. Magnetic bead-bound complexes with AGO2 were immobilized, and unbound material was washed off six times; after digesting proteins with Proteinase-K, the RNAs were extracted for quantitative real-time PCR and AGE (agarose gel electrophoresis) analyses.

### Xenograft assays

Ten BALB/c athymic nude mice (female, 4–6 weeks old and 16–20 g) were purchased from Hubei Research Center of Laboratory Animals (Wuhan, China). All animal experiments were carried out in accordance with the Guide for the Care and Use of Laboratory Animals of Wuhan University. Each mouse was subcutaneously injected with 5 × 10^6^ HCT116 cells on the right flank region. And the liposomal clodronate was injected intravenously for macrophage depletion [27]. After 8 days, the transplanted nude mice were randomly divided into two groups (*n* = 5 each), miR-195-5p agomir or miR agomir NC (RiboBio, Guangzhou, China) was directly injected into the implanted tumor at the dose of 2 nmol/50 μL PBS, and THP1-induced macrophages were injected into the caudal veins at the dose of 10^6^ cells/50 μL per mouse every 3 days for eight times. Tumor dimension was measured at indicative time points. After 29 days, the weights and volumes of tumors were analyzed. One milliliter of blood was gathered via cardiac puncture into EDTA-containing tubes per mouse. The xenograft tumor and blood were collected for further experiments.

### CTC capture

The mice blood samples were processed within 24 h of collection. Circulating tumor cells (CTCs) were isolated and identified by an osISET device as previously reported by our group [28]. In brief, 1 mL blood was diluted with the 0.9% sodium chloride solution into 5-mL total volumes, then transferred to ISET tubes with an 8-μm diameter aperture membrane. The samples were filtered by positive pressure from 12 to 20 mmHg through the device tubes. After that, the membranes in the device tubes were stained with Wright’s stain, then the morphology and number were rechecked using an ordinary microscope (BX51-Olympus, Japan).

### Statistical analysis

For comparisons, one-way analyses of variance, Fisher’s exact tests, chi-squared tests, and two-tailed Student’s *t* tests were performed, as appropriate. *P* < 0.05 was considered statistically significant. The results were expressed as the mean ± SD from at least three independent experiments. Kaplan–Meier curves were used to calculate overall survivals, and the differences were analyzed by a log-rank test. All statistical analyses were conducted using the SPSS 20.0 statistical software (SPSS Inc., IL, USA).

## Results

### Integrated analysis confirmed miR-195-5p deregulation in CRC with poor survivals and is concomitant with upregulation of NOTCH2

We have found miR-195-5p in seven datasets with 387 CRC samples and 386 ANT samples [29]. Slattery et al. performed two newly non-coding RNA profiling analyses with 649 pairs and 28 pairs of colon cancer samples [30] (Additional file 2: Table S1). So we merged together to further confirm the downregulation of miR-195 in CRC (Additional file 3: Figure S1a). We conducted target prediction for validated miR-195-5p with high stringency. Target genes were obtained from both prediction algorithms and experimentally supported databases. Furthermore, gene set enrichment analysis (GSEA) revealed that the predicted targets were enriched in many cancer-related functional pathways (such as EMT, P53, and NOTCH pathways), which were positively correlated with CRC (Additional file 3: Figure S1b-d). To further investigate whether miR-195-5p and NOTCH2 correlate with the survivals of the CRC patients, we performed Kaplan–Meier and Cox’s proportional hazards regression model analyses of TCGA-COAD patients. We found that a low miR-195-5p level and high NOTCH2 level were significantly correlated with poor overall survivals (Additional file 3: Figure S1e-f). We next detected the expression of miR-195-5p and NOTCH2 in 30 pairs of human CRC and ANT samples. Similarly, RT-qPCR showed that miR-195-5p was significantly downregulated in CRC compared with ANT (Fig. 1a, b). Relatively, the expression of NOTCH2 protein was upregulated in CRC (Fig. 1c, d), whereas there was no significant difference in Notch2 mRNA between CRC and ANT (data not shown). Of note, the miR-195-5p level was negatively correlated with the NOTCH2 protein level in the tumors as calculated by Pearson’s correlation (*R*^2^ = 0.3837, *P* = 0.0003) (Fig. 1e).

**Fig. 1:** miR-195-5p was downregulated in CRC tumor samples with upregulation of NOTCH2. **a** miR-195-5p expressions in 6 pair CRC samples. **b** miR-195-5p is significantly decreased in primary human CRC tissues compared with ANT. Mean ± SD is shown. Statistical analysis was conducted using Student’s *t* test. **c** The levels NOTCH2 protein in 6 pairs of CRC samples. **d** NOTCH2 protein is significantly increased in primary human CRC tissues compared with ANT. Mean ± SD is shown. Statistical analysis was conducted using Student’s *t* test. **e** Scatter plots showing the negative correlation between miR-195-5p and NOTCH2 protein levels

### miR-195-5p inhibits CRC cell proliferation, clone formation, migration, and invasion in vitro

To assess the role of miR-195-5p in colorectal cancer cells, we first examined the baseline miR-195-5p RNA and NOTCH2 mRNA levels in six cell lines (NCM460, HCT116, SW480, SW620, DLD-1, and HT29) by RT-qPCR (Additional file 3: Figure S1g-h). We found, compared with normal intestinal epithelium cell line (NCM460), a lower expression of miR-195-5p in DLD-1 and other cell lines. HCT116 (lowest level) and DLD-1 (highest level) cells were transfected with miR-195-5p mimic or miR mimic NC (negative control) and miR-195-5p inhibitor or miR inhibitor NC, respectively. The transfection efficiency was assessed by fluorescence microscopy (Additional file 3: Figure S1i). The effects of miR-195-5p on cell proliferation of HCT116 and DLD-1 cells were examined using clone formation assay and EdU immunofluorescence (IF) staining. Clonogenic assay showed that miR-195-5p decreased the clonogenic survivals of HCT116 cells compared with negative control (NC) groups, while miR-195-5p inhibitor-treated HCT116 cells showed a reversed phenotype, so does DLD-1 (Fig. 2a, b). In addition, EdU immunofluorescence staining assay revealed that miR-195-5p inhibited DNA synthesis in two cell lines (Fig. 2c, d). Conversely, the miR-195-5p inhibitor could mitigate this inhibition (Fig. 2c, d).

**Fig. 2:** miR-195-5p inhibits HCT116 and DLD-1 cell proliferation, migration, and invasion in vitro. **a**, **b** Representative photomicrographs and quantifications of clone formation assay in DLD1 and HCT116 cells after transfection with miR-195-5p mimic, miR-195-5p mimic NC, miR-195-5p inhibitor, or miR-195-5p inhibitor NC for 48 h. **c**, **d** Representative photomicrographs and quantifications of EdU immunofluorescence staining assay in DLD1 and HCT116 cells. Bar = 50 μm. **e**, **f** Photomicrographs and quantifications of wound healing assay. Bar = 100 μm. **g** Transwell migration assays of DLD1 and HCT116 cells carrying different miRNAs. Bar = 100 μm. **h** Total number of cells in five fields was counted manually. **i** Transwell invasion assays of DLD1 and HCT116 cells. Bar = 100 μm. **j** Total number of cells in five fields was counted manually. Mean ± SD are shown. Statistical analysis was conducted using one-way ANOVA. *P < 0.05. **P < 0.01. ***P < 0.001

To determine the effect of altered miR-195-5p expression on the migration and invasion of CRC cells, miR-195-5p mimic, inhibitor, and paired negative control transfected CRC cells were wounded by scratching and maintained for 48 h. In the wound healing assay, cell motility was monitored at designated time points after scratches. The miR-195-5p overexpressed cells migrated toward the wound more slowly than the negative control or the miR-195-5p-inhibited cells (Fig. 2e, f). This result was also confirmed by the transwell migration assay. We found that migration abilities of the miR-195-5p overexpressed cells were significantly inhibited (Fig. 2g, h), whereas the migration ability was higher in the miR-195-5p inhibitor groups. In the transwell invasion assay, we found that invasive abilities of the miR-195-5p overexpressed cells were reduced and could be lifted by the miR-195-5p inhibitor on the contrary (Fig. 2i, j). Taken together, miR-195-5p lowers cell motility, migratory, and invasive abilities.

### Altered miR-195-5p affects colon cancer cell EMT by modulating NOTCH2 expression in a post-transcriptional manner

As mentioned earlier, through bioinformatics analysis, we found that miR-195-5p might target NOTCH2, and the expression of NOTCH2 protein and miR-195-5p was negatively correlated (Fig. 1e), which may affect CRC progression. This reminded that miR-195-5p is likely to modulate NOTCH2 translation. A series of experiments of miR-195-5p and NOTCH2 were performed to further understand the underlying mechanism (Fig. 3 and Additional file 4). After transfecting miR-195-5p mimic, inhibitor, and paired NC, the expression of NOTCH2 mRNA was detected by RT-qPCR. Intriguingly, there was not any difference in the expression levels of NOTCH2 mRNA in the groups of cells (Additional file 5: Figure S3a). Subsequently, the NOTCH2 and activated NOTCH2 (Ad-NOTCH2) protein, EMT-related protein E-cadherin, and Vimentin were verified by western blotting (WB) and immunofluorescence (IF). miR-195-5p mimic-treated cells expressed lower NOTCH2 and Ad-NOTCH2 (Additional file 4: Figure S2a, IF) and Vimentin and higher E-cadherin compared to NC groups, whereas higher NOTCH2, Ad-NOTCH2, and Vimentin and lower E-cadherin were detected in miR-195-5p inhibitor-treated cells (Fig. 3a, b, WB, and Additional file 4: Figure S2b, IF). The results suggest that miR-195-5p negatively regulates NOTCH2, Ad-NOTCH2, and Vimentin levels in CRC cells, while E-cadherin was positively regulated by miR-195-5p, suggesting negative regulations of miR-195-5p on the NOTCH2 pathway and EMT in CRC cells.

**Fig. 3:** miR-195-5p affects colon cancer cell EMT by modulating NOTCH2 expression in a post-transcriptional manner. Western blots of NOTCH2, Ad-NOTVH2, and EMT markers Vimentin and E-Cadherin in DLD1 and HCT116 cells transfected with different miRNAs (**b**) and quantifications of NOTCH2 protein (**c**). Assays were performed in triplicates. A schematic representation of the pmiR-RB-REPORTTM dual-luciferase reporter vector with 3′-UTR of Notch2 mRNA harbors two miR-195-5p cognate sites (**d**). Relative luciferase activity of reporter plasmids carrying wild-type or mutant Notch2 3′-UTR in DLD1 and HCT116 cells co-transfected with miR-195-5p mimic or mimic negative control (mimic NC) (**e**). Notch2 mRNA decay curves of HCT116 cells carrying miR-195-5p mimic or mimic NC (**f**). The decay model was fit in a one-phase exponential decay model. AGO2-RNA immunoprecipitation assay (RIP) showing that miR-195-5p interacted with NOTCH2 in HCT116 cells (**g**). (**P < 0.01, ***P < 0.001)

To confirm the direct regulation of miR-195-5p on NOTCH2 expression, the dual-luciferase reporter assay was carried out. We cloned the NOTCH2 3′-UTR into a luciferase reporter plasmid. NOTCH2 harbors two conserved miR-195-5p cognate sites (44–50 and 1275–1281 of NOTCH2 3′-UTR, Fig. 3c), which were predicted targets of miR-195-5p. The luciferase reporter vector pmiR-RB-REPORTTM-NOTCH2 3′-UTR or mutant reporter vector carrying point mutations of the putative miR-195-5p binding sites was co-transfected with miR-195-5p mimics or mimic NC, separately. The results indicate that miR-195-5p inhibits the luciferase activity in wild-type NOTCH2 3′-UTR transfected HCT116 and DLD-1 cells (Fig. 3d, *P* < 0.05), whereas it did not influence the activity of luciferase in carrying mutant NOTCH2 3′-UTR vector cells. These results suggested that miR-195-5p binds directly to NOTCH2 3′-UTR regions of two predicted binding sites.

We further analyzed the specific role of miR-195-5p for NOTCH2 expression. HCT116 cells were added with actinomycin D after 24 h after being transfected with miR-195-5p mimics or mimic NC. Then the NOTCH2 mRNA levels were detected at designated time points. The NOTCH2 mRNA levels were normalized by GAPDH, and the decay model was fit in a one-phase exponential decay model [31]. The half-lives of miR-195-5p and mimic NC transfected cell mRNA were 4.098 h and 5.102 h (Fig. 3e, no significance), which revealed that miR-195-5p did not affect NOTCH2 mRNA stability. Then AGO2-RNA immunoprecipitation assay (RIP) was performed. There was no difference in the AGO2 protein expression levels of miR-195-5p mimic and mimic NC groups (Additional file 5: Figure S3b, no significance). NOTCH2 mRNA was strongly enriched in the AGO2 immunoprecipitates compared with negative control IgG immunoprecipitates (Fig. 3f). And the miR-195-5p-treated group enriched more NOTCH2 mRNA compared with the NC group (Fig. 3f). Taken together, our results revealed that miR-195-5p might inhibit CRC cell EMT though binding to the NOTCH2 3′-UTR region and suppressing the NOTCH2 protein in a post-transcriptional manner.

### Facilitation of miR-195-5p inhibitor in CRC cell clone formation, proliferation, migration, and invasion is abrogated by silencing NOTCH2

We also assessed the carcinogenicity of NOTCH2 in CRC cells. Three siRNAs (Notch2-homo-1815, 2501 and 3130) were transfected to HCT116 cell, and the expressions of NOTCH2 mRNA and protein were detected with RT-qPCR and WB (Additional file 5: Figure S3c-d). The best siRNA (Notch2-homo-2501) was applied in subsequent experiments. Loss of NOTCH2 expression also contributed to inhibition of CRC cell clone formation (Fig. 4a, b), DNA synthesis (Fig. 4c, d), migration (Fig. 4e, f), and invasion (Fig. 4g, h). As previously mentioned, miR-195-5p inhibitor can facilitate CRC cell clone formation, DNA synthesis, proliferation, migration, and invasion. However, after silencing NOTCH2, the miR-195-5p inhibitor could not play the above role. Moreover, after NOTCH2 was overexpressed by the pGV219 vector, the abilities of CRC cell clone formation, DNA synthesis, migration, and invasion were enhanced (Additional file 6: Figure S4c-f). These effects could be partly abrogated by miR-195-5p mimic. Taken together, these results further confirmed the powerful carcinogenicity of NOTCH2 in CRC and indicated that the anticancer efficacy of miR-195-5p may be partly attributed to its suppressive role on NOTCH2.

**Fig. 4:** Silenced NOTCH2 abrogates the role of the miR-195-5p inhibitor in CRC cell clone formation, proliferation, migration, and invasion abilities. Representative photomicrographs (**a**) and quantifications (**b**) of clone formation assay in HCT116 cells after transfection with the si-NOTCH2, miR-195-5p inhibitor, or si-NOTCH2 together with the miR-195-5p inhibitor for 48 h. Representative photomicrographs (**c**) and quantifications (**d**) of EdU immunofluorescence staining assay. Bar = 50 μm. Transwell migration assays of transfected HCT116 cells (**e**). Bar = 100 μm. Total number of cells in five fields was counted manually (**f**). Transwell invasion assays of HCT116 cells (**g**). Bar = 100 μm. Total number of cells in five fields was counted manually (**h**). Mean ± SD are shown. Statistical analysis was conducted using one-way ANOVA. *P < 0.05. **P < 0.01. ***P < 0.001.

### miR-195-5p inhibits M2-like TAM polarization by suppressing the NOTCH2/GATA3/IL-4 pathway in CRC cells

Focusing on tumor cells and M2-like TAMs in TME, we detected NOTCH2 and CD163 expression and distribution in the CRC and paired ANT tissues of two CRC patients by immunofluorescence. NOTCH2 (red) was highly expressed in CRC tissues (Fig. 5a), especially the invasive tumor front (ITF; white dashed, Additional file 7: Figure S5a), whereas it was lowly expressed in adjacent normal tissues. Interestingly enough, the CD163 (green) expression was concentrated in the invasive tumor front, rather than the tumor nest (Fig. 5a, Additional file 7: Figure S5a). Moreover, miR-195-5p was negatively related with the expression of NOTCH2 and CD163 in CRC and ANT (Fig. 5a). These results might hint that high expression of NOTCH2 can recruit macrophages to ITF and induce M2 polarization, as several studies have shown that NOTCH2 was capable of enhancing IL-4 production though promoting GATA3 expression in mast cells or T cells [22, 32]. However, the mechanism of NOTCH2 inducing IL-4 production in CRC and whether affecting TAM polarization was rarely understood. To verify the hypothesis that NOTCH2 signaling enhances GATA3-mediated IL-4 production in CRC cells, we tested the expression of NOTCH2, GATA3, and IL-4 in patients’ tumor tissues and transfected CRC cells. For two patients, NOTCH2, GATA3, and endogenous IL-4 were strongly expressed and positively correlated in cancer tissues, whereas these were weakly expressed in ANT (Fig. 5b). The results were also confirmed in immunohistochemical staining serial sections (Additional file 7: Figure S5b). In CRC cells, inhibition of miR-195-5p increased the protein levels of NOTCH2, GATA3, and IL-4, but miR-195-5p mimic did abrogate these effects (Fig. 5c). Moreover, after silencing NOTCH2, relative expressions of GATA3 and endogenous IL-4 were decreased (Fig. 5). Comparatively, the levels of GATA3 and endogenous IL-4 were increased after NOTCH2 overexpression (Additional file 6: Figure S4a). Exocrine IL-4 levels in all cell supernatants were further detected by ELISA. The IL-4 level in the miR-195-5p inhibitor group was higher than that in the paired control group, while the IL-4 levels in the miR195-5p mimic-treated, si-NOTCH2, and IL-4 inhibitor (Suplatast Tosilate, IPD 1151 T, a cytokine inhibitor which can inhibit IL-4 expression by cells) groups were lower than those in the negative control groups (Fig. 5e). Moreover, mesenchymal cell lines (SW480 and SW620) expressed higher IL-4 compared to epithelial cell lines (HT29, HCT116, and DLD-1) (Additional file 8: Figure S6a). In conclusion, these results suggested that miR195-5p-mediated IL-4 production relied on the NOTCH2/GATA3/IL-4 signaling pathway in CRC.

**Fig. 5:** miR-195-5p inhibits M2-like TAM activation and recruitment. **a** Fluorescent probe in situ hybridization (FISH) experiment to demonstrate the distribution of miR-195-5p, NOTCH2, and CD163. **b** Western blots of NOTCH2, Ad-NOTCH2, GATA3, and IL-4 of CRC tissues, miR-195-5p-transfected HCT116 (**c**), and si-NOTCH2 or IL-4 inhibitor-treated HCT116 (**d**). **e** ELISA detected the IL-4 levels in cell supernatants. **f**–**i** RT-qPCR tested the macrophage-associated markers after being co-cultured with transfected HCT116. Assays were performed in triplicates. Mean ± SD is shown. Statistical analysis was conducted using one-way ANOVA. *P < 0.05. **P < 0.01. ***P < 0.001

To elucidate whether miR195-5p-mediated IL-4 in CRC cells affects macrophage alternative polarization, co-culture and migration assay of macrophages and CRC cells were performed. After being cultured with transfected CRC cell-conditioned medium, macrophages were inclined to the M2 phenotype (CD163^high^ CD80^low^ IL-10^high^ TGF-β^high^) in the miR-195-5p inhibitor-treated group compared to the inhibitor NC (Fig. 5f, g). After adding IL-4 neutralizing antibody (Anti IL-4) in medium of the miR-195-5p inhibitor-treated group (miR-195-5p + Anti IL-4 group), this effect has disappeared. In the miR-195-5p mimic-treated groups, macrophages seemed to be M1-like (CD163 ^low^ IL-10 ^low^) (Fig. 5f, g). With silenced NOTCH2 or inhibited IL-4 expression by IL-4 inhibitor, macrophages tended to be M1 activated (CD80^high^ CD163^low^ IL-10^low^TGF-β^low^) and downregulation of CD163 (RT-qPCR and FCM, Fig. 5h, i, Additional file 6: Figure S4c-d). These results indicated that IL-4 from CRC cells may be the reason of M2-like TAM polarization. In addition, through wound healing and co-culture cell migration assay, we found that miR-195-5p inhibitor-treated cancer cells would like to favor macrophages while miR-195-5p mimic, si-NOTCH2, and IL-4 inhibitor reversed it (Additional file 8: Figure S6b-g). All in all, our finding indicated that miR195-5p-mediated IL-4-related M2-like TAM polarization and recruitment were a function of the NOTCH2-GATA3-IL-4 signaling pathway in CRC.

### miR-195-5p suppresses tumor growth and M2-like TAM polarization in vivo

To further explore the role of miR-195-5p in vivo, we performed a xenograft nude mouse experiment via subcutaneously injecting HCT116 cells. We found that miR-195-5p upregulation significantly delayed tumor growth (Additional file 8: Figure S6h). And the tumor weights were also decreased on the 29th day post injection after miR-195-5p accumulation (Additional file 8: Figure S6i-j). Furthermore, EMT abilities of formed tumors derived from miR-195-5p-upregulated tumor cells were also impaired (Fig. 6a, b). These results confirmed the suppressing role of miR-195-5p in tumor progression. More importantly, the proposed regulations of miR-195-5p on the expression of NOTCH2, GATA3, and IL-4 in miR-195-5p-agomir-treated tumors were similar to the in vitro results, which substantiated the suppressor function of miR-195-5p in the NOTCH2/GATA3/IL-4 pathway inducing TAM recruitment and M2 polarization (Fig. 6a, b). Since the tumor EMT program may promote CTC generation, we had detected CTCs from blood of every mouse using blood film and CTC capture technology. CTCs were further identified by immunofluorescence staining (Fig. 6d) that miR-195-5p suppressed CTC generation (Fig. 6c, d). Summarily, our research showed that miR-195-5p inhibited the NOTCH2 signaling pathway leading to suppression of EMT and CTCs. miR-195-5p/NOTCH2-mediated IL-4 secretion during CRC EMT is responsible for M2-like TAM polarization.

**Fig. 6:** miR-195-5p suppresses tumor growth and M2-likeTAM infiltration in vivo. **a** Immunohistochemistry of tumor tissues treated with or without miR-195-5p. **b** Western blots of E-cadherin, Vimentin, NOTCH2, Ad-NOTCH2, GATA3 and IL-4 in the tumors. GAPDH was used as a loading control. **c** Representative photomicrographs and quantifications (**d**) of CTCs captured from blood of mice. Assays were performed in triplicates. Mean ± SD is shown. Statistical analysis was conducted using Student’s *t* test. **f** Interaction between CRC EMT and M2-like TAMs in TME

## Discussion

In this study, we found that tumor cells undergoing EMT could secrete IL-4 to activate macrophages to a M2-like phenotype, and dysregulation of miR-195-5p mediated EMT status of CRC cells by regulating NOTCH2. miR-195-5p is a vital role in CRC EMT-related TAM alternative activation and is associated with good prognosis in colorectal tumor patients.

Integrated analysis has been used to identify differentially expressed genes at the mRNA and miRNA in tumors. We had found the downregulation of miR-195-5p in CRC by analyzing seven studies which included 376 paired samples before [29]. However, the more qualified studies included, the higher the reliability of the results will be. So we further assessed the role of miR-195-5p in CRC by incorporating two new studies with 677 paired samples. Above all, reduced expression of miR-195-5p in primary CRC was correlated with poor overall survivals, suggesting that miR-195-5p can be an effective diagnostic and prognostic marker in the clinical setting. Secondly, altered expression of miR-195-5p in colon cancer cell lines considerably modulated cell growth, migration, and invasion. Thirdly, miR-195-5p directly regulated expression of NOTCH2 in a post-transcriptional manner by targeting its 3′-UTR. Finally, miR-195-5p/NOTCH2 modulated IL-4 secretion in CRC to affect M2-like TAM polarization.

miR-195-5p is a member of evolutionarily conserved miRNAs termed the miR-15/107 family which has been suggested to have considerable potential in prognostic prediction [33–35]. miR-195-5p acts as a tumor suppressor in tumor progression by targeting numerous genes, such as YAP1 in CRC [29], RPS6KB1 in prostate cancer [35], MMP14 in cervical carcinoma [36], and NOTCH2 in osteosarcoma [12]. So the rescue experiment is needed to investigate the role of miR-195-5p in the NOTCH2 pathway. Importantly, we showed that after NOTCH2 knockdown in CRC cells, the inhibiting effects of miR-195-5p on EMT progression and cell invasion were partially abrogated. Thus, we propose that downregulation of miR-195-5p in CRC enhanced EMT by deregulating NOTCH2. Similarly, Jin and colleagues also found that miR-195-5p could overcome CRC stemness and chemoresistance by inhibiting NOTCH2 and RBPJ [26]. So miR-195-5p/NOTCH2 may play a crucial role in CRC EMT and progression.

Recent studies have showed that the Notch pathway was involved in tumor EMT [16, 18–20, 37]. The overexpression of NOTCH2 has been observed in numerous human cancer types, such as non-small cell lung cancer [19], gastric carcinoma [20], and CRC [38]. Maraver et al. had revealed that the Notch pathway affected the process of epithelial–mesenchymal transition through its effector HES1 targeting Vimentin promoter in bladder cancer [18]. Intriguingly, they also found the overexpression of ZEB2 after the Notch was inhibited or HES1 was downregulated, even though HES1 did not bind to the ZEB2 promoter observably. Moreover, our previous study also revealed that ZEB2 is downregulated after miR-195-5p upregulation [29]. However, ZEB2 is not a predicted target of miR-195-5p or YAP1, so there may be another regulation between miR-195-5p and ZEB2. Inspired by Maraver’s work, our finding of miR-195-5p/NOTCH2-mediated CRC EMT may be partly contributed by ZEB2. Further investigation is needed to elucidate regulation of NOTCH2 to ZEB2 in CRC EMT.

On the other hand, the NOTCH2 pathway is necessary for IL-4 production [22, 39]. Peng had found that NOTCH2 mediated the initiation of Th2 cytokines (such as IL-4 and IL-5) in Th2 cells through GATA3 [21]. Zhu and colleague proved that GATA3 was required for in the initiation of Il4 transcription during Th2 cell differentiation with a conditional knockout of a Gata3 mouse model [40]. And Tanaka further confirmed that DNase I–hypersensitive site 2 (HS2) element situated in the second intron of the IL-4 locus as a critical enhancer was strictly controlled by GATA-3 binding [22]. Their work had preliminarily illustrated the role of NOTCH2/GATA3 in IL-4 production in Th2 cells. However, the mechanism of IL-4 secretion in CRC is still unclear. In this work, we show that NOTCH2 induced tumor cell EMT status, resulting in the secretion of IL-4 to promote M2 polarization of TAMs. Additionally, after silencing NOTCH2, the expressions of GATA3 and IL-4 were decreased, whereas inhibited IL-4 production by the inhibitor did not decrease levels of NOTCH2 and GATA3. These might indicate that there is a NOtCH2/GATA3/IL-4 axis in CRC cells to affect TAM polarization.

TAMs have been widely recognized as a favorable condition for tumor progression, including tumor cell growth, EMT, and immune suppression in TME. In TME, TAMs were mixed with the M1/M2 phenotype, which may play opposite roles in CRC progression [41–43]. Numerous studies tended to M2-like (CD163^high^ CD80^low^ IL-10^high^ TGF-β^high^) TAMs, which were closely related to poor prognosis of CRC [44]. In this study, THP1-induced macrophages became CRC-conditioned TAMs after incubation with transfected colon tumor cells or cell supernatant. The resultant TAMs displayed characteristics of M2-like macrophages, with CD163^high^, CD80^low^, IL-10^high^, TGF-β^high^, and IL-10^high^ phenotypes. Conversely, after silencing NOTCH2 and inhibiting IL-4, TAMs seemed to be an M1-like phenotype (CD163^low^, CD80^high^, and TGF-β^low^). In TME, M2-like TAMs, which infiltrate into the tumor invasive front, secreted multiple cytokines such as IL-10, TGF-β, and IL-13, to suppress the immune reaction, stimulate angiogenesis and EMT, and remodel ECM [10]. The crucial role of M2-like TAMs in CRC EMT has been preliminarily determined. Reversely, our data showed that EMT-programmed tumor cells produced high levels of IL-4, sequentially causing the increase of M2-like TAM recruitment and polarization in vitro and in vivo. Silenced NOTCH2 and inhibited IL-4 could reduce M2-like TAMs. So these results demonstrated that different tumor cells’ EMT status could affect IL-4-related M2-like TAM polarization. Numerous studies focused on the role of TAMs in tumor progression [11, 41, 43, 45], and rare studies are concerned about tumor EMT status affecting TAM polarization [4, 14]. Our results firstly indicated that miR-195-5p/NOTCH2 regulated IL-4 expression while modulating the EMT of tumor cells, thereby promoting TAM polarizations. It is likely to become a new therapeutic target in CRC.

## Conclusion

In summary, our study suggested that NOTCH2 activation enhanced CRC EMT and NOTCH2/GATA3-mediated IL-4 secretion, ultimately promoting M2-like TAM polarization. miR-195-5p, as a tumor suppressor, directly regulated NOTCH2 expression to inhibit CRC EMT and M2-like TAM polarization. The miR-195-5p/NOTCH2-GATA3/IL-4 axis could be a potential therapeutic target for CRC progression.

## Additional files

Additional file 1: Supplemental experimental procedures. (DOCX 34 kb)

Additional file 2: **Table S1.** Datasets used in finally integrated analysis. (DOCX 18 kb)

Additional file 3: **Figure S1.** (a) miR-195-5p was downregulated in tumor of nine CRC miRNA expression datasets. (b) Gene Set Enrichment Analysis (GSEA) of miR-195-5p targeted genes were enriched in NOTCH pathway and positively related in CRC (*P* = 0.049). (c) miR-195-5p targeted genes were enriched in P53 pathway (*P* = 0.009). (d) Targeted genes of miR-195-5p were enriched in EMT-related pathway (*P* < 0.001). (e) Kaplan–Meier plots for overall survivals for median miR-195-5p expression, from TCGA sequencing data to assess prognostic accuracy. *P* values were calculated using the log-rank test. (f) Kaplan–Meier plots for overall survivals from TCGA sequencing data for median Notch2 expression. P values were calculated using the log-rank test. (g) miR-195-5p expression in six cell lines. (f) NOTCH2 expression in six cell lines. (i) Transfection efficiency of miR-195-5p was assessed by fluorescence microscopy. (PDF 7526 kb)

Additional file 4: **Figure S2.** (a) Immunofluorescence detected the expression of NOTCH2 in transfected cells. (b) Immunofluorescence detected the expression of E-cadherin and Vimentin in transfected cells. (PDF 835 kb)

Additional file 5: **Figure S3.** (a) RT-qPCR analyzed the Notch2 mRNA of transfected HCT116 cells. (ns = No Significant difference). (b) Western blots of AGO2 protein in miR-195-5p mimic and mimic NC groups for RIP assay. (c) Relative expression of Notch2 mRNA in HCT116 cells transfected with three siRNAs. (d) Western blots of NOTCH2 protein in in HCT116 cells transfected with three siRNAs. (e) miR-195-5p relative expression after altered NOTCH2. (f) Western blot analysis of expression of NOTCH2 and Ad-NOTCH2. (PDF 268 kb)

Additional file 6: **Figure S4.** (a) Western blot analysis of expression of NOTCH2, Ad-NOTCH2, GATA3, IL-4 and E-cadherin and Vimentin. (b) ELISA about supernatant from NOTCH2 overexpression with/without miR-195-5p mimic. (c) Clone formation assay. (d) EdU immunofluorescence staining. (e) Transwell migration assay. (f) Transwell invasion assay. (PDF 1779 kb)

Additional file 7: **Figure S5.** (a) Tumor nest overexpressed NOTCH2 (red) with more CD163+ (green) TAM infiltration in invasive tumor front (ITF, white dashed) compared with ANT of three representative CRC patients by immunofluorescence staining. (b) Immunohistochemical staining serial sections of CRC tissues. (PDF 7783 kb)

Additional file 8: **Figure S6.** (a) ELISA detected the IL-4 levels in supernatants of five cells. (b) Quantifications of CD163+ ratios of macrophages co-cultured with si-NOTCH2 or IL-4 inhibitor-treated HCT116 cells. (c) Flow cytometry detected CD163 of macrophages co-cultured with si-NOTCH2 or IL-4 inhibitor-treated HCT116 cells. (d) Representative photomicrographs and quantifications (e) of Ibidi-wound healing assay of macrophages and miRNAs-treated HCT116. Bar = 100 μm. Transwell migration assays of macrophages (f). Bar = 100 μm. Total number of cells in five fields was counted manually (g). Assays were performed in triplicates. Mean ± SD is shown. Statistical analysis was conducted using one-way ANOVA. *P < 0.05. **P < 0.01. ***P < 0.001. (h) Photographs of the mice that were treated with miR-195-5p Agomir or NC. (i) Weights and photographs of dissected tumors. (j). Tumor volume growth curves. (PDF 1982 kb)

## Abbreviations

ANT: Adjacent normal tissue
CRC: Colorectal cancer
CTCs: Circulating tumor cells
EMT: Epithelial–mesenchymal transition
RIP: RNA immunoprecipitation
TAMs: Tumor-associated macrophages
TME: Tumor microenvironment
